# Image Enhancement Model Based on Deep Learning Applied to the Ureteroscopic Diagnosis of Ureteral Stones during Pregnancy

**DOI:** 10.1155/2021/9548312

**Published:** 2021-10-29

**Authors:** Xiao-Yan Miao, Xiao-Nan Miao, Li-Yin Ye, Hong Cheng

**Affiliations:** ^1^Department of Radiation Oncology, The First People's Hospital of Fuyang (Fuyang First Affiliated Hospital of Zhejiang Chinese Medical University Ben Giang College), Hangzhou, China 311400; ^2^Department of Endocrinology, The First People's Hospital of Fuyang (Fuyang First Affiliated Hospital of Zhejiang Chinese Medical University Ben Giang College), Hangzhou, China 311400; ^3^Department of Urology, The First People's Hospital of Fuyang (Fuyang First Affiliated Hospital of Zhejiang Chinese Medical University Ben Giang College), Hangzhou, China 311400; ^4^Department of Ultrasound, The First People's Hospital of Fuyang (Fuyang First Affiliated Hospital of Zhejiang Chinese Medical University Ben Giang College), Hangzhou, China 311400

## Abstract

**Objective:**

To explore the image enhancement model based on deep learning on the effect of ureteroscopy with double J tube placement and drainage on ureteral stones during pregnancy. We compare the clinical effect of ureteroscopy with double J tube placement on pregnancy complicated with ureteral stones and use medical imaging to diagnose the patient's condition and design a treatment plan.

**Methods:**

The image enhancement model is constructed using deep learning and implemented for quality improvement in terms of image clarity. In the way, the relationship of the media transmittance and the image with blurring artifacts was established, and the model can estimate the ureteral stone predicted map of each region. Firstly, we proposed the evolution-based detail enhancement method. Then, the feature extraction network is used to capture blurring artifact-related features. Finally, the regression subnetwork is used to predict the media transmittance in the local area. Eighty pregnant patients with ureteral calculi treated in our hospital were selected as the research object and were divided into a test group and a control group according to the random number table method, 40 cases in each group. The test group underwent ureteroscopy double J tube placement, and the control group underwent ureteroscopy lithotripsy. Combined with the ultrasound scan results of the patients before and after the operation, the operation time, time to get out of bed, and hospitalization time of the two groups of patients were compared. The operation success rate and the incidence of complications within 1 month after surgery were counted in the two groups of patients.

**Results:**

We are able to improve the quality of the images prior to medical diagnosis. The total effective rate of the observation group was 100.0%, which is higher than that of the control group (90.0%). The difference between the two groups was statistically significant (*P* < 0.05). The adverse reaction rate in the observation group was 5.0%, which was lower than 17.5% in the control group. The difference between the two groups was statistically significant (*P* < 0.05). The comparison results are then prepared.

**Conclusions:**

The image enhancement model based on deep learning is able to improve medical diagnosis which can assist radiologists to better locate the ureteral stones. Based on our method, double J tube placement under ureteroscopy has a significant effect on the treatment of ureteral stones during pregnancy, and it has good safety and is worthy of widespread application.

## 1. Introduction

To study the problem of medical image enhancement, it is necessary to have a comprehensive and accurate understanding of its related models, related theories, and current research status, so as to complete the modeling of image enhancement. In this paper, we mainly focus on the research of medical image deblur enhancement technology and underwater medical image enhancement technology. This paper is mainly divided into two parts. As for medical image deblur enhancement technology, we mainly introduce medical deep learning based on a convolutional neural network model. The deep learning model is the main model of medical image deblur enhancement technology, and the color theory and color balance are applied in the medical image enhancement method proposed by us. This paper uses this method to study the application of deep learning in ureteral calculi during pregnancy.

Ureteral stones are one of the most common diseases in urology, and it is not uncommon in clinical work for ureteral stones to progress to urosepsis. Such patients have a rapid onset, rapid progress, and a dangerous condition. Some patients even have systemic inflammatory response syndrome even before the hospital admission. The vital signs have been unstable. If they are not treated promptly and correctly, the condition will quickly get out of control and deteriorate. The case fatality rate is as high as 22%-76%. Pregnant women often develop urinary calculi due to changes in endocrine status in the body, but considering the safety of mothers and infants, conservative medical treatment is often used; for pregnant women who do not respond to medical treatment, appropriate surgical procedures for gravel are very important to ensure the safety of mothers and infants [1].

The incidence of ureteral stones during pregnancy is about 0.026% to 0.0531%. The incidence of menopausal women is higher than that of primiparous women, with an average age of 27 years [2–4]. The incidence during pregnancy is almost the same as that during nonpregnancy, with a ratio of 1 : 1500 to 1 : 200 [5]. 80% to 90% of patients have stone-related clinical manifestations in the second trimester (13 to 27 weeks of gestation) and the third trimester (28 to 40 weeks of gestation) [6–9], and stone-related clinical manifestations in the first trimester (1 to 12 weeks of pregnancy) are rare. Changes in special physiological anatomy during pregnancy lead to a higher incidence of stones on the right than on the left, and calcium phosphate stones are more common [10]. Although the incidence of ureteral stones during pregnancy is relatively low, renal colic caused by ureteral stones is the main reason for nonobstetric hospital admission during pregnancy [11]. The diagnosis and treatment of ureteral stones during pregnancy are special and complicated and often require joint diagnosis and treatment of multiple departments. In the diagnosis and treatment of patients with ureteral stones during pregnancy, the safety of pregnant women and fetuses must be considered. Because radiation (CT) has a clear detrimental effect on fetal development, it is not recommended as a routine diagnosis and treatment technique for urinary stones during pregnancy. Ultrasound examination has no damage to fetal development, so it can be used as a first-line method for diagnosing ureteral stones. Most patients with symptomatic ureteral stones during pregnancy can be relieved by conservative treatments such as spasmolysis, analgesia, and anti-infection. However, for patients with unsatisfactory results of conservative treatment, surgical intervention should be actively given to minimize the potential harm of surgery on pregnant women and fetuses and surgical stimulation-induced threatened abortion.

Ultrasound is a sound wave with a frequency higher than 20000 Hz. It has good directivity and strong reflection ability, and it obtains more concentrated acoustic energy easily. The propagation distance in water is farther than that in air. It can be used for distance measurement, speed measurement, cleaning, sterilization, etc. There are many applications in medicine. Ultrasound is named because its lower frequency limit exceeds the upper limit of human hearing. The working principle of medical ultrasound examination is similar to that of sonar; that is, the ultrasound is emitted into the human body. When it meets the interface in the body, it will reflect and refract, and it may be absorbed and attenuated in human tissue. Because the shape and structure of various tissues of the human body are different, the degree of reflection and refraction and absorption of ultrasonic waves are also different. Doctors are distinguishing by the characteristics of the wave mode, curve, or image reflected by the instrument.

In recent years, the number of patients with ureteral calculus obstruction has also increased in recent years. Ureteral calculi obstruction disease itself will not have a great impact on pregnancy, but complications such as urinary tract infections caused by stones may cause premature delivery or even miscarriage.

For patients with ureteral calculi obstruction in late pregnancy, minimally invasive surgery should be taken in time. In the diagnosis and treatment of patients with ureteral calculi during pregnancy, the safety of pregnant women and fetuses must be considered. Because radiation (CT) has a clear detrimental effect on fetal development, it is not recommended as a routine diagnosis and treatment technique for urinary stones during pregnancy. Ultrasound examination has no damage to fetal development, so it can be used as a first-line method for diagnosing ureteral stones. Most patients with symptomatic ureteral stones during pregnancy can be relieved by conservative treatments such as spasmolysis, analgesia, and anti-infection. However, for patients who are not satisfied with conservative treatment, surgical intervention should be actively given to minimize the potential harm of surgery on pregnant women and fetuses and surgical stimulation-induced threatened abortion.

## 2. Materials and Methods

### 2.1. Image Enhancement Based on the Regional Neural Network

#### 2.1.1. Overview of Image Deblur and Enhancement Methods

In order to improve the effect and stability of the blurring artifact removal and enhancement work, to obtain blurring artifact-free images with complete details and saturation and contrast restored, and to improve the efficiency of the work, we introduce the convolutional neural network model into the blurring artifact removal and enhancement work. By establishing the relationship between the media transmittance and the image with blurring artifacts, the model can estimate the media transmittance map of each region in the image with blurring artifacts. In order to preserve the integrity of the restored blurring artifact-free image in detail, we also added the detail enhancement operation. In order to enable the operation to complete the autonomous parameter adjustment, we combined this method with the evolutionary algorithm and proposed the evolution-based detail enhancement method. The deblur artifact enhancement method proposed is shown in Figure 1, where the left box is the neural network deblur artifact model, which is used to estimate the media transmittance of the input image with blurring artifacts and the right box is the blurring artifact removal and enhancement image. The left box part is the detail enhancement part, which carries out the detail enhancement operation on the image after the blurring artifact removal enhancement.

#### 2.1.2. Deblurring and Identification of Ureteral Stones in Images Using Region-Based Neural Networks

The region-based neural network model of blurring artifact removal takes the blur images as input and outputs the media transmissivities of blurring artifacts, in which each point corresponds to a local region in the input image. In our design, the neural network model is a full convolution structure, as shown in Figure 2.

The network structure consists of a feature extraction network and a regression subnetwork. The feature extraction network is used to capture blurring artifact-related features in the input image, while the regression subnetwork is used to predict the media transmittance in the local area. In order to connect the two network structures, each position on the N-channel feature map output by the feature extraction network will be transmitted to the sliding windows of the c1 group, and the size of each sliding window is 3 × 3. For each sliding window, the output is a feature vector in dimension c1, and each feature vector corresponds to a local region in the input image with blurring artifacts. Then, all the eigenvectors are mapped to a set of features in c2 dimension by a set of 1 × 1 convolution. Obtain the final prediction of the ureteral stone predicted map. The connection between the sliding window and the local region of the blurring artifact image is called the anchor connection. The corresponding local region in the input image can be regarded as the anchor point, and the media transmittance in an anchor point can be approximately a constant. The process is described as follows:

(1) $$\begin{array}{c} \overset{\sim }{t}\left(p\right)=F\left(I\left(i\right)\right),{iIw}_{r}\left(P\right), \end{array}$$

where *F* is the deblur artifact neural network model, which takes blurring artifact image I as its input. $\overset{\sim }{t}\left(p\right)$ is the value of transmittance in the *R*∗*R* region centered on *P*.

## 3. Feature Extraction through the Convolutional Neural Network

In this stage, the network structure is mainly composed of two basic network units, which are used to extract relevant features from input images.

1. We designed and integrated multiple levels of features. The input *x* is passed through two separate branches, and the outputs of these branches are then recombined. The specific operation can be expressed as follows:

(2) $$\begin{array}{c} y_{a}=f\left(x\right)+g\left(x\right), \end{array}$$

(3) $$\begin{array}{c} f\left(x\right)=W_{\left|x\right|}*\theta \left(W_{3*3}*\theta \left(x\right)\right), \end{array}$$

(4) $$\begin{array}{c} g\left(x\right)=W_{\left|x\right|}*\theta \left(W_{\left|x\right|}*x\right), \end{array}$$

where *W*_1×1_ and *W*_3×3_ represent 1 × 1 and 3 × 3 convolution kernels, respectively.

Specifically, *f*(*x*) is a convolutional neural network structure based on heterogeneous convolutional kernels, which are composed of 3 × 3 and 1 × 1 convolutional layers. Among them, 1 × 1 convolution operation can capture more details of blurring artifacts, while 3 × 3 convolution operation can better extract the overall distribution features of blurring artifacts.

(2) A module has a residual structure. Networks with residual modules are easier to optimize and can achieve better performance as the number of layers of the network model increases as defined as follows:

(5) $$\begin{array}{c} y_{b}=f\left(x\right)+x, \end{array}$$

where *y*_*b*_ represents the underlying mapping and *f*(*x*) is a residual mapping constructed by stacking nonlinear layers.

### 3.1. Patient Information

Eighty pregnant patients with ureteral stones treated in the urology department of our hospital from December 2018 to October 2019 were selected as the research subjects, and all patients met the diagnostic criteria of pregnancy with ureteral stones [12–14]. Exclusion criteria were as follows: suffering from pregnancy combined with hypertension, diabetes, etc.; combined with severe organic and mental diseases such as heart, liver, kidney, and other organs; and combined with other surgical contraindications. Patients and their families signed an informed consent form.

The study was approved by the hospital ethics committee and was filed by the medical department. All patients were divided into the test group and control group according to random number table method, 40 cases in each group. The age of the test group was 24 years to 39 years, the average age was 29.31 ± 3.65 years, the gestational week was 5 weeks to 35 weeks, and the average was 28.63 ± 5.64 weeks. Among them, there were 12 cases in the early pregnancy, 17 cases in the middle period, and 11 cases in the late period; in the control group, the age was 25-40 years, the average age was 29.41 ± 3.55 years, the gestational week was 5 weeks to 36 weeks, and the average was 28.71 ± 5.58 weeks, including 11 cases in early pregnancy, 19 cases in the midterm, and 10 cases in the late period. There was no statistically significant difference in the basic conditions such as age and gestational age between the two groups (*P* > 0.05), and they were comparable.

### 3.2. Treatment Method

All patients were given symptomatic treatment such as antispasmodic and analgesic after admission. Patients with lower urinary tract infection were treated with conventional anti-infective treatment. Before the operation, routine care was performed [15–17]. Progesterone was injected intramuscularly 20 minutes before the operation. The experimental group underwent cystoscopy double J tube placement: the patient took the bladder lithotomy position for local anesthesia of the urethral mucosa, and we placed the cystoscope through the urethral opening, looked for stones under the endoscope, and guided the guidewire to guide the ureteral opening into the 6F double J tube, and observed the urine drainage situation and routine postoperative B-ultrasound to confirm the placement of the double J tube. The images were then further improved in terms of better resolution and quality by our proposed image enhancement and deblur technique. The control group underwent ureteroscopy lithotripsy: the patient took the bladder lithotomy position and received epidural anesthesia after routine disinfection. A ureteroscope was placed through the urethral orifice, under the guidance of the guidewire into the affected ureter, and a lithotripsy probe was inserted. Continuous pulses are used to crush stones, and the size of the stones does not exceed 3 mm. Large stones can be removed by foreign body forceps, and double J catheters are routinely placed. All patients had double J catheters removed through ureteroscopy 4 weeks after surgery and were given routine anti-infective and symptomatic treatment after surgery.

### 3.3. Observation Index

Comparing the operation time, time to get out of bed, and hospitalization time of the 2 groups of patients, the operation success rate of the 2 groups of patients and the incidence of complications within 1 month after surgery were counted. Reexamination of B-ultrasound 1 month after the operation revealed that the diameter of the remaining stones was <3 mm, and the patient's symptoms such as nausea, vomiting, and hematuria disappeared, indicating successful operation.

### 3.4. Statistical Method

SPSS19.0 statistical software was used to process the data. The measurement data was expressed as *x* ± *s*, the *t*-test was used, the count data was expressed as a percentage, and the *X*^2^ test was used. *P* < 0.05 means that the difference was statistically significant.

## 4. Results

### 4.1. Comparative Analysis

As shown in Figure 3, the original images (Figure 3(a)) are improved by our proposed image enhancement and deblur technique, which results in images (Figure 3(b)) with better resolution and quality.

### 4.2. Comparative Analysis of Medical Images

In order to make the treatment of ureteral stones during pregnancy with double J tube placement under ureteroscopy better and more obvious, this study selected two sample patients for in-depth study and demonstration, which we denote as subject 1 and subject 2.  Figure 4 is an ultrasound scan image of subject 1, and Figure 5 is an ultrasound scan image of subject 2. Note that this image comparison is performed after performing denoising and deblur.

### 4.3. Comparison of Treatment Effect

The total effective rate of the observation group was 100.0%, which is higher than that of the control group (90.0%). The difference between the two groups was statistically significant (*P* < 0.05). The treatment situation is shown in Table 1. The statistical graph of treatment effect is shown in Figure 6.

### 4.4. Comparison of Adverse Reactions

The adverse reaction rate in the observation group was 5.0%, which was lower than 17.5% in the control group. The difference between the two groups was statistically significant (*P* < 0.05). The comparison results are shown in Table 2.

## 5. Discussion

Ureteral calculi and renal colic during pregnancy are two of the common emergencies for nonobstetric causes of pregnant women. The incidence of ureteral stones in pregnant women is reported to be from 0.04% to 0.5% [18]. Decreased estrogen levels during pregnancy will lead to increased blood calcium, while increased progesterone levels will cause ureteral smooth muscle tension to decrease, thicken the wall, and reduce peristalsis, which will increase the probability of stones staying in the ureter. In addition, the enlarged uterus during pregnancy and the right-handed uterus will also compress the ureter, resulting in obstruction of urinary flow and dilation of the ureter. It is also an important factor that induces the formation of stones and affects the discharge of stones [19, 20]. However, renal colic, urinary tract obstruction, and urinary tract infections caused by ureteral stones during pregnancy may cause miscarriage and premature delivery of pregnant women, and timely and effective treatment is urgently needed. For patients with ureteral calculi during pregnancy with small stone diameters and mild symptoms, conservative treatment can be tried first, including anti-infection, antispasmodic analgesia, and hydration. Some ureteral stones can be discharged by themselves.

Due to changes in hormone levels and physiological structure in pregnant women, ureteral stones are a common disease of pregnant women. In addition to the current dietary changes, the incidence of ureteral stones has also increased year by year. Pregnancy combined with ureteral stones has often multiple stones, which is easy to cause urinary tract obstruction and severe pain. If it is not diagnosed in time and no appropriate treatment is taken, it will cause patients with hydronephrosis [21–23]. Clinical treatment of pregnancy combined with ureteral calculi often adopts conservative medical methods. For patients who do not respond to medical treatment, two surgical methods cystoscopy double J tube placement and ureteroscopy lithotripsy are commonly used [24, 25]. The purpose of this study is to compare the clinical effects of these two surgical methods in the treatment of pregnancy with ureteral stones and to provide a reference for clinical treatment.

In recent years, the incidence of ureteral calculi obstruction has increased in the second and third trimesters of pregnancy. Patients have symptoms such as dysuria, pain, and even hematuria [26, 27]. Mainly due to the increase in kidney circulation during pregnancy, it leads to an increase in water-soluble vitamins in patients' urine, which leads to urinary tract infection [28]. It has also been suggested in the study that an excessively large uterus may also cause compression of the ureter, making it difficult for stones to be expelled. And in recent years, it has been clinically proposed that the incidence of ureteral calculi obstruction in the second and third trimesters of pregnancy is also affected by factors such as physiological changes in pregnant women during pregnancy. For patients with ureteral stone obstruction in the second and third trimesters of pregnancy, early treatment can improve the patient's prognosis and reduce the incidence of adverse pregnancy outcomes. Clinically, ureteroscopy double J tube placement, ballistic lithotripsy, etc. are commonly used in the treatment of late pregnancy with ureteral calculi obstruction, but the effect after ballistic lithotripsy is not satisfactory, and the stone removal rate is low, so the residual stones are more common. And there are many postoperative complications, which are easy to cause urinary tract infection and affect the prognosis [29].

This paper shows that the operation time of the experimental group with double J tube placement under cystoscopy was significantly shorter than that of the control group, but the hospitalization time was significantly longer than that of the control group; there was no difference in the average time to get out of bed and the success rate of surgery between the two groups.

And there were no postoperative complications. The purpose of surgical treatment of ureteral stones is to relieve urethral obstruction, thereby alleviating the symptoms. The improved ultrasound scans in terms of image quality can assist the radiologists to better locate the ureteral stones. Ureteroscopic lithotripsy is the first surgical method for clinical treatment of ureteral calculi because of its simple operation, accurate treatment effect, and few postoperative complications. It is widely used in clinic, and the surgical method is relatively mature [30]. It can manually adjust the ultrasonic amplitude to ensure the safety of the mother and baby, the treatment time is short, and the hospitalization cost can be reduced. Cystoscopy double J tube placement is a new surgical method that has emerged with the rapid development of material technology in recent years. Some studies have shown that its treatment of pregnancy with ureteral calculi has a significant effect and not only can relieve urinary tract obstruction but also can effectively reduce the renal pelvis. Internal pressure can also drain urine, thereby reducing the risk of infection. Double J tube placement surgery can avoid ultrasonic lithotripsy, maximize the safety of pregnant women and fetuses, and ensure continued pregnancy. The material of the double J tube is stable, and it is not easy to produce stimulation and rejection reaction to the human body and can be left in the body for a long time. Cystoscopy double J tube placement and ureteroscopy lithotripsy have significant effects and safety in the treatment of pregnancy with ureteral calculi [31]. We also realize that it is important that deep learning-based frameworks [32–34] be implemented to deblur or even segment the regions of interest in the medical images for a better analysis. In summary, cystoscopy double J-tube placement and ureteroscopy lithotripsy have significant effects on pregnancy and ureteral calculi, and they have good safety. The clinical method can be selected according to the patient's wishes and specific circumstances.

## 6. Conclusion

The ureteroscope has the advantages of less trauma and less infection, and if residual gravel is found in the actual lithotripsy treatment or the ureter is twisted, it can be reinserted into the soft ureteroscope to clean it again, which can significantly improve the rate of stone removal and prevent the recurrence of stones. At the same time, the double J tube is placed in the lithotripsy, the lens body and the optical fiber are always unified, and the advantage of treating ureteral stone obstruction is more obvious.

The results of the study show that after ureteroscopy double J tube implantation, the patient's stone removal and drainage are significantly better than those of patients with sinus lithotripsy, suggesting that the treatment effect of ureteroscopy double J tube implantation is more ideal. The results of this study are consistent with this. And in this study, the observation group had a higher success rate of lithotripsy than the control group, and the total adverse reaction rate was lower than that of the control group, suggesting that ureteroscopy double J tube placement surgery has higher safety and successful operation.

According to the influence of medical image quality, we propose the deblur enhancement method and medical image enhancement method, respectively. In medical image enhancement methods to the blurring modeling based on a deep learning problem by a deep neural network model to estimate the blurring image transmission rate of media and through the inverse operation of deep learning, restore clear medical images and put forward a detail enhancement algorithm based on evolutionary finish to restore clear details of medical image enhancement operation. Finally, we apply the simplified deblur model to low computing power.

In summary, combined with medical image deblur techniques and ultrasound scanning, the effect of ureteroscopy double J tube implantation in the treatment of midlate pregnancy with ureteral stone obstruction is ideal, which greatly improves clinical symptoms, promotes recovery, and reduces the incidence of adverse reactions.

## Figures and Tables

**Figure 1:** The deblur and image enhancement method.

**Figure 2:** Region-based neural network model processing flow.

**Figure 3:** Comparison of (a) original and (b) improved images.

**Figure 4:** Ultrasound scan image of ureteral stones in subject 1 ((a) original scan image and (b) postoperative scan image). The arrow points to the location of the ureteral stones. Note that the stones were located much easier by the radiologists after image quality enhancement. This demonstrates that the medical image deblur and denoising algorithms are useful and have strong clinical applicability in accurate medical image diagnosis.

**Figure 5:** Ultrasound scan image of ureteral stones in subject 2 ((a) original scan image and (b) postoperative scan image). The arrows in the medical images point to the ureteral stones, which show up clearly after image enhancement.

**Figure 6:** Statistics of the treatment effect.

**Table 1:** Treatment effect statistics (*n* = 40).

Group	Marked effect	Effective	Invalid	Total efficiency
Observation group	32	8	0	40 (100.0%)
Control group	27	9	4	36 (90.0%)
*X* ^2^	10.384	0.323	11.982	11.982
*P* value	0.001	0.426	0.001	0.001

**Table 2:** Statistics of the occurrence of adverse reactions (*n* = 40).

Group	Bleeding in the vagina	Mild urinary system infection	Abortion	Premature delivery	Total adverse reaction rate
Observation group	1 (2.5%)	1 (2.5%)	0	0	2 (5.0%)
Control group	3 (7.5%)	2 (5.0%)	1 (2.5%)	1 (2.5%)	7 (17.5%)
*X* ^2^	1.094	0.358	1.024	2.093	4.601
*P* value	0.294	0.540	0.311	0.149	0.032

## Data Availability

The image data used to support the findings of this study have been deposited in the renal and ureteral stone dataset (https://www.payititi.com/nlpdataset/show-1437.html).
